# Inhibition of miR-27b Regulates Lipid Metabolism in Skeletal Muscle of Obese Rats During Hypoxic Exercise by Increasing PPARγ Expression

**DOI:** 10.3389/fphys.2020.01090

**Published:** 2020-08-31

**Authors:** Xuebing Wang, Yingli Lu, Lei Zhu, Haibo Zhang, Lianshi Feng

**Affiliations:** ^1^School of Kinesiology, Shanghai University of Sport, Shanghai, China; ^2^College of Physical Education, Guangxi University, Nanning, China; ^3^Exercise Biology Research Center, China Institute of Sport Science, Beijing, China; ^4^School of Sports Science, Qufu Normal University, Qufu, China

**Keywords:** miR-27b, PPARγ, hypoxic exercise, lipid metabolism, skeletal muscle

## Abstract

Hypoxic exercise may represent a novel therapeutic strategy to reduce and prevent obesity through the regulation of lipid metabolism. During hypoxic exercise, the targeting of peroxisome proliferator-activated receptor gamma (PPARγ) by miR-27b has been proposed to be one of the mechanisms involved in the modulation of lipid metabolism. We have previously shown that miR-27b can repress PPARγ and lipid metabolism-associated factors, thereby affecting lipid metabolism during hypoxic exercise in a rat model of obesity. In the current study, we aimed to confirm the role of miR-27b in the regulation of lipid metabolism. First, miR-27b expression was either upregulated or downregulated through the injection of adeno-associated virus (AAV) 9 containing a miR-27b expression cassette or miR-27b-3p inhibitor, respectively, into the right gastrocnemius muscle of obese rats. The rats were then subjected to a 4-week program of hypoxic exercise, and a series of parameters related to lipid metabolism were systematically evaluated, including body composition, blood lipid levels, miR-27b RNA levels, and mRNA and protein levels of PPARγ and those of its downstream lipid metabolism-associated factors. No significant differences were found in body composition between rats expressing different levels of miR-27b. However, regarding blood lipids, miR-27b overexpression led to increased concentrations of triglycerides (TG), low-density lipoprotein cholesterol (LDL-C), and free fatty acids (FFAs), while inhibition of miR-27b decreased the total cholesterol (TC) level and increased that of high-density lipoprotein cholesterol (HDL-C). At the mRNA level, miR-27b overexpression downregulated the expression of *Ppar*γ, but upregulated that of lipid metabolism-associated factors such as heart-type fatty acid-binding protein (H-FABP), fatty acid transport protein 1 (FATP1), adipose triglyceride lipase (ATGL), and lipoprotein lipase (LPL), whereas miR-27b inhibition elicited the opposite effect; however, inhibition of miR-27b led to elevated cholesterol 7 alpha-hydroxylase (CYP7A1) and fatty acid translocase 36 (CD36) levels. Similarly, at the protein level, miR-27b overexpression promoted a decrease in the concentration of PPARγ, whereas miR-27b inhibition led to an increase in PPARγ levels, as well as those of CYP7A1, CD36, ATGL, and LPL. Overall, our results indicated that hypoxic exercise regulates lipid metabolism via the miR-27b/PPARγ pathway and modulates ATGL and LPL expression through inducing their post-transcriptional modifications.

## Introduction

Obesity with weight gain due to the consumption of highly caloric foods has become a worldwide health problem (Park et al., 2019). Obese individuals, in addition to displaying high body weights, also exhibit high weight to height ratios and a risk of dyslipidemia associated with elevated blood lipid levels (Han and Lean, 2016; Camacho-Cardenosa et al., 2019). Regular aerobic exercise is typically recommended for weight loss purposes, as it burns fat as a fuel source. However, an intervention involving only pure exercise may increase appetite, and intensive exercise must usually be undertaken over an extended period (>6 months) for weight loss to occur (Park et al., 2019).

For obese individuals, moving to, and living in, a hypoxic environment can lead to a reduction in body weight. Similarly, hypoxic exercise over a short period can also lead to greater weight loss compared with normoxic exercise (Westerterp and Kayser, 2006; Kayser and Verges, 2013; Kong et al., 2014), which has been associated with the promotion of lipid metabolism during hypoxic training (Workman and Basset, 2012; Yingli et al., 2014; Camacho-Cardenosa et al., 2018b). However, it is critical that the mechanisms and signaling pathways underlying the effects of hypoxic exercise are understood before it can be widely used as a weight-loss strategy in the treatment of obesity and associated comorbidities (Kayser and Verges, 2013).

Lipid metabolism has been well-characterized. MicroRNAs (miRNAs) were recently found to regulate lipid metabolism-related gene expression (Singh et al., 2018). In particular, miR-27b, miR-33, miR-122, and miR-148a have been shown to be involved in regulating lipid metabolism (McGregor and Choi, 2011; Castaño et al., 2018; Xinbo et al., 2018). Importantly, miR-27b was reported to regulate the expression of several crucial lipid metabolism-related transcription factors (Chen et al., 2012), including peroxisome proliferator-activated receptor gamma (PPARγ) (McGregor and Choi, 2011). MiR-27b can bind the 3′UTR of PPARγ mRNA and suppress its expression (McGregor and Choi, 2011). Meanwhile, PPARγ can regulate the expression of a series of lipid metabolism-related genes, including cholesterol 7 alpha-hydroxylase (*CYP7A1*), fatty acid translocase 36 (*CD36*), heart-type fatty acid-binding protein (*H-FABP*), fatty acid transport protein (*FATP*), adipose triglyceride lipase (*ATGL*), and lipoprotein lipase (*LPL*) (Zhu et al., 2015; Hsu et al., 2018; d’Angelo et al., 2019; Xu et al., 2019). Interestingly, both hypoxia and exercise have been reported to modulate the expression levels of miR-27b and PPARγ (Park and Park, 2012; Sutliff et al., 2013; Tomaz et al., 2016). We have also previously shown that hypoxic exercise can enhance lipid metabolism via the miR-27b/PPARγ pathway in obese rats (Yingli et al., 2017; Zhu et al., 2018, 2019). However, it is unclear how miR-27b and PPARγ regulate lipid metabolism to affect weight loss during hypoxic exercise.

In this study, we hypothesized that miR-27b/PPARγ was the key lipid metabolism regulation pathway operating during hypoxic exercise in obese rats. To test this, we utilized adeno-associated virus serotype 9 (AAV9)-mediated up- or downregulation of miR-27b expression in the gastrocnemius muscle of obese rats, and then observed the effect on lipid metabolism following 4 weeks of hypoxic exercise.

## Materials and Methods

### Generation of an Animal Model of Obesity

The protocols used in this study were approved by the Animal Use Committee of the China Institute of Sport Science. A total of 120, 3-week-old male Sprague–Dawley rats weighing 60–90 g each were purchased from Beijing Vital River Laboratory Animal Technology Co., Ltd. and housed under standard specific-pathogen-free (SPF) conditions (12 h light/dark cycle, a temperature of 21–23°C, relative humidity of 40–60%, and free access to food and water). After being given a normal diet (Beijing Vital River Laboratory Animal Technology Co., Ltd.) for 1 week, the rats were randomly assigned to two groups. In one group, the rats continued being fed with a normal diet (Control, *n* = 20), whereas in the other group, the rats were fed with a high-fat diet (HFD, *n* = 100) (D12451, 45% energy from soybean oil and lard; Research Diets, United States), for 10 weeks. A HFD-fed rat was considered to be obese if its body weight exceeded the average body weight of the Control rats by 20% (Yang et al., 2012; Ji et al., 2016). The overweight rats were excluded compared with the average weight of obese rats. Finally, 50 obese rats were then subjected to 2 weeks of an adaptive treadmill exercise. The exercise speed was gradually increased from 16 to 20 m/min, and the duration of the exercise from 20 to 60 min/day, over 2 weeks. During 2-week adaptive training, individual performance of 50 obese rats was recorded in daily training. The performance included if the animal can complete the planned training intensity and training time. According to the individual performance records, 40 of the 50 obese rats were selected and randomly divided into four groups of 10 rats each for AAV9 delivery and hypoxic exercise (see below) (Figure 1).

**FIGURE 1:** Flow chart describing the generation of a rat model of obesity and animal experiments.

### AAV9 Vector Production

The strategy for the construction of the transgene-containing plasmid used for packaging AAV9-ZsGreen-rno-miR-27b and that for packaging the AAV9-ZsGreen-rno-miR-27b-3p inhibitor is shown in Tables 1, 2. Briefly, rat miR-27b and the miR-27b-3p inhibitor were synthesized and amplified. Then, miR-27b and the inhibitor were cloned into the pAAV9-ZsGreen vector to construct pAAV9-ZsGreen-rno-miR-27b and the pAAV9-ZsGreen-rno-miR-27b-3p inhibitor, respectively. The transgene-containing plasmids pAAV9-ZsGreen-rno-miR-27b, pAAV9-ZsGreen-rno-miR-27b-3p, and pAAV9-ZsGreen were co-transfected with helper plasmids into 293T AAV cells to generate AAVs. After 3 days, the cells were collected and lysed by repeated cycles of freezing and thawing at −80 and 37°C, respectively, to acquire recombinant AAVs (rAAV9s). rAAV9s were purified using the ViraBind^TM^ AAV9 Purification Mega Kit (VPK-141, Cell Biolabs) (Li et al., 2019). The virus titer was measured by qPCR (Li et al., 2019) and adjusted to 1 × 10^12^ viral genomes (vg)/mL.

**TABLE 1:** Construction of a transgene-containing plasmid for packaging AAV9-ZsGreen-rno-miR-27b.

Gene name	rno-mir-27b MI0000859
Cloning vector	pAAV-ZsGreen-miRNA
Cloning strategy	*Bam*HI + *Eco*RI
Synthesized rno-miR-27b (5′→3′)	GGATCCACCTCTCTAACAAGGT GCAGAGCTTAGCTGATTGGTGAAC AGTGATTGGTTTCCGCTTTGT TCACAGTGGCTAAGTTCTGC ACCTGAAGAGAAGGTGGAATTC

**TABLE 2:** Construction of a transgene-containing plasmid for packaging AAV9-ZsGreen-rno-miR-27b-3p inhibitor.

Gene name	rno-miR-27b-3p MIMAT0000798
Cloning vector	pAAV-ZsGreen-shRNA
Cloning strategy	*Bam*HI + *Hin*dIII
miR-27b-3p-inhibitor-F (5′→3′)	GATCCGCAGAACTTCAGACTGTGAACGCG GCAGAACTTCAGACTGTGAATTTTTTA
miR-27b-3p-inhibitor-R (5′→3′)	AGCTTAAAAAATTCACAGTCTGAAGTTCTGCC GCGTTCACAGTCTGA

*F, forward primer; R, reverse primer.*

### Intramuscular Injection of rAAV9 Into Obese Rats

Before subjecting the obese rats to hypoxic training, rAAV9 was delivered into the gastrocnemius muscle of each tested obese rat by intramuscular injection. Five injection sites were chosen in the right gastrocnemius muscle and 10 μL of rAAV9 (1 × 10^12^ vg/mL) was injected into each site. AAV9-ZsGreen was delivered to 10 obese rats assigned to the placebo control group (C), AAV9-ZsGreen-miR-27b to 10 obese rats assigned to the mir-27b overexpressing group (O), and AAV9-ZsGreen-miR-27b-3p inhibitor to 10 obese rats assigned to the mir-27b inhibition group (I). The remaining 10 uninjected obese rats were assigned to the hypoxic sedentary group (H) (Figure 1).

### Model for Training Under Hypoxic Conditions

The four groups of obese rats were housed under hypoxic conditions with 13.6% O_2_. The rats in groups C, O, and I were made to exercise on a treadmill at a speed of 20 m/min for 1 h/day, 5 days/week, for a total of 4 weeks; the rats in group H were not made to exercise. After the final training session, the rats in groups C, O, and I were allowed to recover for 24 h (Figure 1). Then, the rats from all the groups were fasted for 12 h, after which body length and weight were measured. The body mass index (BMI) and Lee’s index were calculated via the following formulas: Body mass index (BMI) = body weight/length (cm)^2^; and Lee’s index = body weight (g)^1/3^/body length (cm) × 1000. The rats were then euthanized by intraperitoneal injection of a 10% (0.3 mL/100 g) trichloroacetaldehyde hydrate solution and quickly fixed on an ice-covered sampling board. Between 5 and 7 mL of blood was collected from the abdominal aorta and placed in coagulant-containing tubes. Serum was separated by centrifuging the blood in the tubes (3,000 rpm, 10 min) and stored at −20°C. The left perirenal and epididymal fat pads were quickly separated and weighed and the right gastrocnemius muscle was collected and frozen at −80°C.

### Blood Lipid Level Measurement

Frozen serum samples were thawed to measure the concentrations of blood lipids, including total cholesterol (TC), triglyceride (TG), low-density lipoprotein cholesterol (LDL-C), high-density lipoprotein cholesterol (HDL-C), and free fatty acids (FFAs), using commercially available kits (TC, TG, HDL-C, LDL-C: Prodia Diagnostics, Germany; FFAs: Nanjing Jiancheng Bioengineering Institute, China) (Zhou et al., 2013).

### RNA Extraction and Quantitative Reverse Transcription PCR (RT-qPCR)

MiR-27b expression levels and the mRNA levels of lipid metabolism-related genes were determined by RT-qPCR. First, total RNA was extracted from gastrocnemius muscle using Trizol (Invitrogen, United States) and treated with DNase I (Fermentas, United States). Then, cDNA was obtained by reverse transcription of the isolated RNA using M-MLV reverse transcriptase (Takara, Dalian, China), dNTPs (Takara, Dalian, China), and RNase Inhibitor (Fermentas). The synthesized cDNA was used as a template for follow-up experiments or stored at −80°C.

qPCR primers for RNAs (miR-27b and *U6*) (Table 3) and cDNAs (beta-actin, *Ppar*γ, *Cyp7a1*, *Cd36*, *Atgl*, *H-Fabp*, *Lpl*, and *Fatp1*) (Table 4) were designed and synthesized by Tianyi Huiyuan Biotechnology, Beijing, China. qPCR was performed in an Applied Biosystems 2720 thermal cycler using SYBR Premix Ex Taq (Takara). Each sample was analyzed three times. *U6* was used as the housekeeping gene for miR-27b and beta-actin was used for the other genes. The ΔΔC_*T*_ method was used to quantify relative expression levels (Livak and Schmittgen, 2001).

**TABLE 3:** Primers used in the RT-qPCR analysis of miR-27b.

Gene	Primer sequence (5′→3′)	Length (nt)
miR-27b	RT:CTCAACTGGTGTCGTGGAGTCGGC AATTCAGTTGAGCTGTTC	42
	F: GGCGACCAGAGCTTAGCTGAT	21
	R: CTCAACTGGTGTCGTGGAGTC	21
*U6*	RT: CGCTTCACGAATTTGCGT	18
	F: CTCGCTTCGGCAGCACA	17
	R: CGCTTCACGAATTTGCGT	18

*RT, primer for reverse transcription; F, forward primer; R, reverse primer; nt, nucleotides.*

**TABLE 4:** Primers used for RT-qPCR analysis of lipid metabolism-related genes.

Gene	Primer sequence (5′→3′)	Amplicon size (bp)
Beta-actin	F: GAAGTGTGACGTTGACATCCG	282
	R: GCCTAGAAGCATTTGCGGTG	
*Ppar*γ	F: CTGCGTCCCCGCCTTAT	181
	R: TTCAATCGGATGGTTCTTCG	
*Cyp7a1*	F: GGTTGGAAGAAGCGAACACTGGAT	141
	R: CAGGAATGTGGGCAGCGAGAAC	
*Cd36*	F: GTCCTATTGGGAAAGTTATTGCG	214
	R: TGGGTTCTGGAGTGGGGAG	
*H-Fabp*	F: TGACCAAGCCGACCACAATCATT	150
	R: TCACGACCGACTTGACCTTCCT	
*Fatp1*	F: AGGTTGCTGTGGTGTTCTCTTGG	162
	R: TGGCTTGGTGGCTGAGGTGA	
*Atgl*	F: GGATGAAGGAGCAGACAGGTAGC	134
	R: TGGCACAGACGGCAGAGACT	
*Lpl*	F: CGCTCCATCCATCTCTTCATTGAC	168
	R: GCTTCTCTTGGCTCTGACCTTGT	

*F, forward primer; R, reverse primer.*

### Western Blot Assay

Lipid metabolism-related protein expression was detected using western blot assays. First, total protein was isolated from the gastrocnemius muscle. Specifically, the frozen tissue was cut into small pieces, 20 mg of which was added to 200 μL of protein lysis buffer (Solarbio, China); the mixture was then homogenized on ice using a glass grinder. The homogenate was transferred to a pre-cooled 1.5 mL Eppendorf tube and placed on ice for 15 min for complete lysis. Subsequently, the mixture was centrifuged at 12,000 rpm for 10 min and the supernatant collected and frozen at −20°C. Protein concentration was measured using a BCA protein quantification kit (Cwbiotech, Beijing, China). A total of 30 μg of protein was loaded and separated by electrophoresis, transferred to a PVDF membrane, blocked with 5% BSA–TBST, and incubated overnight at 4°C with the following primary antibodies: mouse anti-rat PPARγ (1:1,000; ab41928, Abcam), mouse anti-rat CYP7A1 (1:500; MABD42, Millipore), mouse anti-rat CD 36 (1:1,000; MABT399, Millipore), rabbit anti-rat ATGL (1:2,000; ab109251, Abcam), rabbit anti-rat H-FABP (1:200; ab45966, Abcam), mouse anti-rat LPL (1:500; MABS1270, Millipore), and rabbit anti-rat FATP1 (1:1,000; PA5-67913, Invitrogen). After washing three times with TBST, the membrane was incubated for 1 h at room temperature with horseradish peroxidase (HRP)-conjugated goat anti-rabbit IgG (H + L) (Jackson, #111-035-003) or HRP-conjugated goat anti-mouse IgG (H + L) (Jackson, #115-035-003) secondary antibodies (1:10,000 dilution). After washing three times with TBST, enhanced chemiluminescence (ECL) reagent (WBKLS0500, Millipore) was added to the protein surface of the membrane followed by incubation for 3 min at room temperature. The membrane was developed for 2 min and then fixed. The gray values of target proteins were analyzed using Image-Pro Plus 6.0 image software (Media Cybernetics, Georgia, United States).

### Spontaneous Fluorescence of a Frozen Section of Gastrocnemius Muscle

To confirm the successful delivery of rAAV9 into the gastrocnemius muscle, we determined whether ZsGreen was expressed alone or with miR-27b in the gastrocnemius muscles of group C, O, and I rats. First, frozen gastrocnemius muscle was embedded with optimal cutting temperature (OCT) compound (#4583, Sakura), refrozen at −70°C, and solidified. Then, serial sections were obtained using a freezing microtome (Thermo, CRYOSTAR NX50). Finally, the tissue sections were observed and imaged under a fluorescence microscope (MS23).

### Statistical Analysis

All statistical analyses were performed using SPSS 17.0 (IBM). Comparisons between two groups were performed using one-way ANOVA and LSD tests. Data were presented as means ± standard deviation (SD). A *p*-value < 0.05 was considered statistically significant.

## Results

### A Rat Model of Obesity Was Generated by Feeding Rats With a High-Fat Diet for 10 Weeks

Rats in the HFD and Control groups were fed for 10 weeks with, respectively, a HFD and a normal diet. The body weight of the rats was measured weekly (Figure 2). After 10 weeks, the average body weight of the HFD-fed rats was 24% greater than that of the Control rats (610.0 ± 32.3 g vs. 490.0 ± 26.7 g), indicating that the HFD could induce obesity. After adaptive exercise, 40 obese rats were selected for use in subsequent experiments.

**FIGURE 2:** The body weight of rats fed a high-fat diet (HFD; *n* = 100) and of those fed a normal diet (Control, *n* = 20) was measured weekly for 10 weeks. Data are presented as means ± SD.

### AAV9 Was Successfully Delivered Into the Gastrocnemius Muscle of Obese Rats

After 4 weeks of hypoxic exercise, the efficiency of AAV9 transfection and the miR-27b expression level in the gastrocnemius muscle were assessed (Figures 3, 4). Under the fluorescence microscope, the tissue sections from the rats in groups O, I, and C appeared green, while the tissue sections from the uninjected rats in group H were dark (Figure 3). Furthermore, RT-qPCR analysis indicated that, compared with rats in the C and H groups, the relative miR-27b expression level increased in the rats from group O and decreased in those from group I (Figure 4). Additionally, the mean miR-27b level was similar between rats in group C and those in group H (Figure 4). These results confirmed that rAAV9 was successfully delivered and efficiently transduced into gastrocnemius muscle.

**FIGURE 3:** Representative fluorescence images of the gastrocnemius muscle of rats injected with AAV9-ZsGreen-miR-27b (group O), AAV9-ZsGreen-miR-27b-3p inhibitor (group I), or AAV9-ZsGreen (group C), as well as of rats not injected with AAV9 (group H). The gastrocnemius muscle of rats in groups O, I, and C show ZsGreen fluorescence. Tissue sections of frozen gastrocnemius muscle were obtained using a freezing microtome and observed under a fluorescence microscope. Scale bar = 500 μm.

**FIGURE 4:** The expression levels of miR-27b relative to those of *U6* in obese rats from groups O, I, C, and H measured by RT-qPCR. Results were compared by one-way ANOVA; all data are presented as means ± SD. **p < 0.01.

### Hypoxic Exercise Reduced the Weights and Other Body Composition Indexes of Obese Rats

The body weight, fat weight (epididymis fat weight plus perirenal fat weight), BMI, and Lee’s index of the four groups are shown in Table 5. After 4 weeks of hypoxic exercise, the body weight, fat weight, BMI, and Lee’s index of the obese rats in groups C, O, and I were significantly decreased compared with those of the sedentary rats from group H (Table 5). In addition, there was no significant difference between the body composition indexes of the rats of groups C, O, and I, except that the mean epididymal fat weight of the rats in group I was higher than that of the rats in group C (Table 5).

**TABLE 5:** Effects of hypoxic training on the body composition of obese rats.

	Group O	Group I	Group C	Group H
Body weight before hypoxic exercise (g)	631.1 ± 31.5	629.2 ± 31.9	630.3 ± 31.6	641.9 ± 33.7
Body weight after hypoxic exercise (g)	561.8 ± 27.3**	559.0 ± 39.7**	534.4 ± 48.3**	704.6 ± 56.2
Perirenal fat weight (g)	1.94 ± 0.67**	2.16 ± 0.69*^#^	1.38 ± 0.63**	2.90 ± 0.66
Epididymal fat weight (g)	4.84 ± 1.79**	5.09 ± 1.45**	4.17 ± 1.37**	8.24 ± 2.30
BMI	7.71 ± 0.32**	7.60 ± 0.64**	7.24 ± 0.42**	9.20 ± 0.49
Lee’s index	305.63 ± 6.26**	303.60 ± 10.43**	298.71 ± 5.22**	321.56 ± 7.50

Results were compared by one-way ANOVA; all data are presented as means ± SD. *p < 0.05, **p < 0.01, vs. the rats in group H; ^#^p < 0.05, vs. the rats in group C. BMI, body mass index.

### Both Hypoxic Exercise and miR-27b Expression Levels Affected Blood Lipid Concentrations in Obese Rats

Table 6 shows the mean levels of TC, TG, HDL-C, LDL-C, and FFAs. Compared with the rats in group H, the levels of TG, LDL-C, and FFAs were significantly decreased (all *p* < 0.01) in rats of the I, O, and C groups (Table 6). Furthermore, compared with the rats in group C, those in group O displayed higher levels of TG and LDL-C (*p* < 0.05 and *p* < 0.01, respectively), while rats in group I exhibited significantly lower TC levels (*p* < 0.05) and higher HDL-C levels (*p* < 0.01). Compared with rats in group O, the concentrations of TC, TG, LDL-C, and FFAs in rats of group O were all markedly decreased (all *p* < 0.01), whereas those of HDL-C were greatly increased (*p* < 0.01).

**TABLE 6:** Serum lipid levels measured in all the groups of obese rats.

Blood lipids (mmol/L)	Group O	Group I	Group C	Group H
TC	1.64 ± 0.20	1.20 ± 0.20^#&&^	1.45 ± 0.12	1.61 ± 0.161
TG	0.70 ± 0.04**^#^	0.48 ± 0.10**^&&^	0.58 ± 0.06**	0.87 ± 0.12
HDL-C	0.44 ± 0.04	0.62 ± 0.05**^##&&^	0.50 ± 0.06**	0.40 ± 0.07
LDL-C	0.66 ± 0.06**^##^	0.44 ± 0.08**^&&^	0.52 ± 0.06**	0.83 ± 0.12
FFA	0.57 ± 0.04*	0.49 ± 0.03**^&&^	0.52 ± 0.08**	0.63 ± 0.06

Results were compared by one-way ANOVA; all data were presented as means ± SD. *p < 0.05, **p < 0.01, vs. the rats in the group H; ^#^p < 0.05,^ ##^p < 0.01, vs. the rats in group C; ^&&^p < 0.01, vs. the rats in group O. TC, total cholesterol; TG, triglyceride; HDL-C, high-density lipoprotein cholesterol; LDL-C, low-density lipoprotein cholesterol; FFA, free fatty acids.

### Both Hypoxic Exercise and miR-27b Regulated the Expression of PPARγ and Its Downstream Lipid Metabolism Regulators at Both the mRNA and Protein Levels

The mRNA and protein levels of the lipid metabolism-related gene *Ppar*γ and those of its downstream genes are shown in Figures 5A,B.

**FIGURE 5:** The expression of the lipid metabolism regulator PPARγ and that of its downstream effectors (CYP7A1, CD36, H-FABP, FATP1, ATGL, and LPL) were determined at the mRNA level by RT-qPCR **(A)** and at the protein level by western blot assays **(B)** in obese rats housed under hypoxic conditions, undergoing hypoxic training, and with regulated miR-27b expression. O: obese rats with overexpression of miR-27b and undergoing hypoxic training; I: obese rats with suppressed miR-27b expression and undergoing hypoxic training; C: obese rats undergoing hypoxic training only; and H: obese sedentary rats without regulation of miR-27b expression. Results were compared by one-way ANOVA; all data are presented as means ± SD. *p < 0.05, **p < 0.01.

Compared with the rats in group H, those in group C displayed higher mRNA levels of *Cd36* and *Atgl* (*p* < 0.05 and *p* < 0.01, respectively), and a lower mean expression level of *Cyp7a1* (*p* < 0.01); the CD36 and ATGL protein levels were similar between these two groups. In the rats from group O, compared with those in group H, the mRNA levels of *H-Fabp*, *Fatp1*, *Cd36*, *Atgl*, and *Lpl* were increased (*p* < 0.05, *p* < 0.01, *p* < 0.01, *p* < 0.05, and *p* < 0.05, respectively) and those of *Ppar*γ and *Cyp7a1* decreased (both *p* < 0.01). Meanwhile, in the rats from group I, both the mRNA and protein levels of PPARγ, CYP7A1, and CD36 were increased compared with those in group H (mRNA level: *p* < 0.01, *p* < 0.01, *p* < 0.05; protein level: *p* < 0.05, *p* < 0.05, *p* < 0.01); the mRNA levels of *Fatp1*, *Atgl*, and *Lpl* were downregulated (*p* < 0.01, *p* < 0.05, and *p* < 0.05, respectively), while the protein levels of ATGL and LPL were significantly increased (both *p* < 0.01) (Figures 5A,B).

Compared with the rats in group C, those from group O displayed a lower mean *Ppar*γ mRNA level (*p* < 0.01) and higher mean *H-Fabp*, *Lpl*, and *Fatp1* mRNA levels (*p* < 0.05, *p* < 0.05, and *p* < 0.01, respectively); the protein concentrations were similar between the O and C groups. Rats from group I (miR-27b inhibition) displayed higher PPARγ, CYP7A1, and CD36 mRNA and protein levels (mRNA level: *p* < 0.01, *p* < 0.01, and *p* < 0.01; protein level: *p* < 0.05, *p* < 0.05, and *p* < 0.01), reduced *Fatp1* and *Atgl* mRNA levels (both *p* < 0.01), and increased ATGL and LPL protein levels (both *p* < 0.01) (Figures 5A,B).

Furthermore, compared with rats from the miR-27b overexpression group (group O), those with downregulated miR-27b expression (group I) exhibited increased mRNA and protein levels of PPARγ, CYP7A1, and CD36 (all *p* < 0.01), reduced mRNA levels of *H-Fabp*, *Fatp1*, *Atgl*, and *Lpl* (*p* < 0.01, *p* < 0.01, *p* < 0.05), and higher ATGL and LPL protein levels (both *p* < 0.01) (Figures 5A,B).

## Discussion

Being obese is becoming the new normal worldwide. Reducing food intake and doing physical exercise are effective and economical ways of preventing or treating obesity. However, physical exercise can also lead to increased appetite and a longer intervention time before weight loss occurs (Park et al., 2019). Recent studies have reported that hypoxia can suppress appetite, and training under hypoxic conditions can reduce fat and weight in a shorter period (Westerterp and Kayser, 2006; Kayser and Verges, 2013; Kong et al., 2014), which was also confirmed in our previous studies (Yingli et al., 2017; Zhu et al., 2018, 2019). We further found that miR-27b contributes to the regulation of lipid metabolism by modulating the expression of PPARγ and lipid metabolism-related genes in the liver and skeletal muscle of obese rats (Yingli et al., 2017; Zhu et al., 2018, 2019). In the current study, to clarify the role of miR-27b in the regulation of lipid metabolism in obese rats subjected to hypoxic exercise, AAV9-ZsGreen-miR-27b and AAV9-ZsGreen-miR-27b-3p inhibitor were employed to upregulate or downregulate miR-27b expression in the gastrocnemius muscle of obese rats, respectively (Figures 3, 4). After 4 weeks of hypoxic exercise, we assessed the body composition, blood lipid levels, and expression levels of miR-27b, PPARγ, and PPARγ-regulated lipid metabolism-related genes, with the results revealing that changes in miR-27b expression levels could modulate lipid metabolism in obese rats subjected to hypoxic exercise.

Recent studies have shown that hypoxic training can reduce body weight and body fat in humans and rodents (Ji et al., 2017; Camacho-Cardenosa et al., 2018a; Yang et al., 2018; Park et al., 2019; Wang et al., 2019). This effect might be due to hypoxic exercise leading to the suppression of appetite (Matu et al., 2017). Similarly, in the present study, hypoxic exercise (13.6% O_2_) for 4 weeks improved the body composition of obese rats, including increasing weight loss and fat loss, as well as lowering BMIs and Lee’s indexes (Table 5). However, our data also indicated that AAV9-mediated changes in miR27b expression in the gastrocnemius muscle of obese rats did not affect the body composition parameters of this muscle when the obese rats were exposed to hypoxic exercise, indicating that mir-27b expression in skeletal muscle may not exert a direct effect on weight and fat loss (Table 5).

Several human and animal studies have shown that hypoxic exercise can improve obesity-related blood lipid parameters (Ling et al., 2008; Shin, 2015; Can et al., 2016; Matu et al., 2017). Here, we also found that hypoxic exercise could decrease TG and LDL-C levels in the blood, while increasing that of HDL-C (Table 6). In order to illustrate the mechanism of the effect of hypoxic exercise on blood lipid, this study observed the changes of miR-27b expression on blood lipids in obese rats with hypoxic exercise. MiR-27b was recently reported to be a key regulator of cholesterol and lipid metabolism (Hsu et al., 2018). In obese people, elevated miR-27 levels in the blood have been associated with higher TG and LDL-C levels and lower HDL-C levels (Can et al., 2016); moreover, it has been suggested that miR-27b can accelerate the development of arteriosclerosis by reducing the expression of PPARγ, thereby inducing perivascular adipose tissue hypertrophy (Chen et al., 2012). In the current work, miR-27b expression in the rat gastrocnemius muscle was precisely controlled by using AAV viral vectors (Figures 3, 4). After 4 weeks of hypoxic exercise, we found that suppressing the expression of miR-27b in the gastrocnemius muscle of obese rats led to a decrease in the serum levels of TC, TG, LDL-C, and FFAs and increased that of HDL-C, consistent with the results of previous studies that showed that inhibition of miR-27b could improve blood lipid levels (Table 6). Conversely, in human hepatoma cells, miR-27b has also been shown to repress cholesterol synthesis, while in zebrafish, miR-27b depletion enhances endotrophic intravascular lipid accumulation in the liver (Selitsky et al., 2015; Hsu et al., 2018). This indicates that the effects of miR-27b on lipid metabolism may differ according to the experimental model used.

Obesity is often accompanied by dyslipidemia (Zhang et al., 2019). Although regular exercise can improve blood lipid composition in obese people, the underlying mechanism is still unclear. Elucidating how blood lipid metabolism is regulated at the molecular level during hypoxic exercise may contribute to the design of guidelines to reduce obesity. PPARγ, a nuclear receptor, has been shown to function as a transcription factor that regulates the expression of lipid metabolism-related genes and, consequently, blood lipid levels (Zhu et al., 2015; d’Angelo et al., 2019), while miR-27b can inhibit PPARγ expression (Hsu et al., 2018). Our data also showed that a negative correlation exists between miR-27b and PPARγ at both the RNA and protein levels (Figure 5).

CYP7A1, an important enzyme for the conversion of cholesterol into bile acids, is a biomarker for reverse cholesterol transport (Chen and Huang, 2009). Several studies have reported that PPARγ regulates the expression of CYP7A1, which suggests that miR-27b/PPARγ/CYP7A1 might comprise a pathway that regulates the metabolism of both cholesterol and polyunsaturated fatty acids (Ge et al., 2017; Han et al., 2019; Luo et al., 2019). Our data demonstrated that elevated PPARγ levels enhanced the mRNA and protein expression of CYP7A1, which may promote the reverse transport of cholesterol in skeletal muscle while lowering the accumulation of total cholesterol in the blood (Figure 5). Consequently, our results support that inhibition of miR-27b and hypoxic exercise can enhance cholesterol metabolism.

In skeletal muscle, oxidation of long-chain fatty acids (LCFAs) supplies most of the energy at rest or during contraction (Koonen et al., 2005). However, owing to the limited storage capability of skeletal muscle, most fatty acids are taken up from the blood by fatty acid transporters (Koonen et al., 2005), including CD36, FATP1, and H-FABP (Koonen et al., 2005; Jain et al., 2009). Of these, CD36 has been shown to be the most efficient at transporting fatty acids, and during prolonged low-intensity exercise, CD36 complexes with carnitine palmitoyltransferase I (CPTI) to enhance LCFA oxidation (Holloway et al., 2006; Schenk and Horowitz, 2006; Nickerson et al., 2009). In addition, CD36 expression is repressed by miR-27b in THP-1 macrophages. However, the 3′UTR of *Cd36* lacks miR-27b binding sites, and a PPARγ expression array analysis further showed that CD36 is a downstream effector of PPARγ (Zhang et al., 2014; Fell et al., 2019), suggesting that miR-27b may indirectly regulate the expression of CD36 through PPARγ. Our findings showed that inhibition of miR-27b expression increased the mRNA and protein levels of CD36 by enhancing PPARγ expression in obese rats undergoing 4 weeks of hypoxic exercise. These results provided novel evidence to support that hypoxic exercise can promote fatty acid oxidation in a miR-27b/PPARγ/CD36 pathway-dependent manner.

MiR-27b/PPARγ pathway can regulate lipid metabolism and both ATGL and LPL are shown to accelerate TG hydrolysis to release fatty acids for oxidation (Schoonjans et al., 1996; Lee et al., 2019). It is reported that miR-27b could inhibit LPL mRNA expression, while PPARγ regulated the mRNA expression of ATGL and LPL (Schoonjans et al., 1996; Kershaw et al., 2007; Karbiener et al., 2009; Lee et al., 2019). Therefore, miR-27b/PPARγ pathway may affect ATGL and LPL mRNA expression, which in turn causes protein expression changes of these genes. However, in this study, we observed that the ATGL and LPL mRNA levels decreased, whereas the ATGL and LPL protein levels increased, after 4 weeks of hypoxic exercise in the gastrocnemius muscle of obese rats with suppressed miR-27b expression and promoted PPARγ expression (Figure 5). The inconsistency between the protein and mRNA expression of ATGL and LPL might be related to post-transcriptional regulation (Hughes, 2006). Several studies have reported that changes in ATGL mRNA and protein expression often show opposing trends, for instance, in the adipose tissue of obese subjects (Steinberg et al., 2007), fasting (Nielsen et al., 2011) or leptin-treated porcine adipocytes (Li et al., 2010). Moreover, acromegaly treatment and improved diabetes control can also result in a difference between LPL mRNA protein level (Simsolo et al., 1992, 1995), and Isoproterenol and insulin could regulate Lpl gene expression by affecting Lpl transcription and steady-state mRNA levels, respectively, suggestive of a post-transcriptional effect (Raynolds et al., 1990). These observations have demonstrated that post-transcriptional regulation of ATGL and LPL may be the common mechanisms that both of them are regulated by some hormones and under certain physiological conditions (Ong and Kern, 1989; Simsolo et al., 1993; Nielsen et al., 2014).

## Conclusion

In conclusion, both hypoxic exercise and inhibition of miR-27b were effective at alleviating the symptoms of obesity, leading to fat and weight loss, decreased levels of TC, TG, LDL-C, and FFAs, and increased levels of HDL-C. Moreover, we showed that the miR-27b/PPARγ pathway regulated the expression of the downstream lipid metabolism-related factors, CYP7A1 and CD36, at both the mRNA and protein levels, and that hypoxic exercise may influence ATGL and LPL expression via post-transcriptional regulation. Overall, our results provided strong evidence for hypoxic exercise being an efficient and effective means of promoting lipid metabolism in obese rats, and may aid healthcare providers in devising reasonable guidelines for the treatment of obesity.

## Data Availability Statement

The raw data supporting the conclusions of this article will be made available by the authors, without undue reservation, to any qualified researcher.

## Ethics Statement

The animal study was reviewed and approved by the animal use committee at the China Institute of Sport Science.

## Author Contributions

XW, LZ, and HZ developed protocols and conducted experiments. XW wrote the manuscript. YL and LF conceived the study, finalized the study design, provided oversight for its conduct, and revised the manuscript. All authors contributed to the article and approved the submitted version.

## Conflict of Interest

The authors declare that the research was conducted in the absence of any commercial or financial relationships that could be construed as a potential conflict of interest.

## References

[B1] Camacho-CardenosaA.Camacho-CardenosaM.Brazo-SayaveraJ.BurtscherM.TimónR.OlcinaG. (2018a). Effects of high-intensity interval training under normobaric hypoxia on cardiometabolic risk markers in overweight/obese women. *High Alt. Med. Biol.* 19 356–366. 10.1089/ham.2018.0059 30204493

[B2] Camacho-CardenosaA.Camacho-CardenosaM.BurtscherM.Martínez-GuardadoI.TimonR.Brazo-SayaveraJ. (2018b). High-intensity interval training in normobaric hypoxia leads to greater body fat loss in overweight/obese women than high-intensity interval training in normoxia. *Front. Physiol.* 9:60. 10.3389/fphys.2018.00060 29472870PMC5810257

[B3] Camacho-CardenosaA.Camacho-CardenosaM.OlcinaG.TimónR.Brazo-SayaveraJ. (2019). Detraining effect on overweight/obese women after high−intensity interval training in hypoxia. *Scand. J. Med. Sci. Sports* 29 535–543. 10.1111/sms.13380 30615248

[B4] CanU.BuyukinanM.YerlikayaF. H. (2016). The investigation of circulating micro RNAs associated with lipid metabolism in childhood obesity. *Pediatr. Obes.* 11 228–234. 10.1111/ijpo.12050 26223376

[B5] CastañoC.KalkoS.NovialsA.PárrizasM. (2018). Obesity-associated exosomal miRNAs modulate glucose and lipid metabolism in mice. *Proc. Natl. Acad. Sci. U.S.A.* 115 12158–12163. 10.1073/pnas.1808855115 30429322PMC6275521

[B6] ChenJ.HuangX. F. (2009). The effects of diets enriched in beta-glucans on blood lipoprotein concentrations. *J. Clin. Lipidol.* 3 154–158. 10.1016/j.jacl.2009.04.054 21291810

[B7] ChenW. J.YinK.ZhaoG. J.FuY. C.TangC. K. (2012). The magic and mystery of microRNA-27 in atherosclerosis. *Atherosclerosis* 222 314–323. 10.1016/j.atherosclerosis.2012.01.020 22307089

[B8] d’AngeloM.CastelliV.TuponeM. G.CatanesiM.AntonosanteA.Dominguez-BenotR. (2019). Lifestyle and food habits impact on chronic diseases: roles of PPARs. *Int. J. Mol. Sci.* 20 5422–5452. 10.3390/ijms20215422 31683535PMC6862628

[B9] FellG. L.ChoB. S.DaoD. T.Anez-BustillosL.BakerM. A.NandivadaP. (2019). Fish oil protects the liver from parenteral nutrition-induced injury via GPR120-mediated PPARγ signaling. *Prostaglandins Leukot. Essent. Fatty Acids* 143 8–14. 10.1016/j.plefa.2019.02.003 30975380PMC6642797

[B10] GeZ.ZhangM.DengX.ZhuW.LiK.LiC. (2017). Persimmon tannin promoted macrophage reverse cholesterol transport through inhibiting ERK1/2 and activating PPARγ both in vitro and in vivo. *J. Funct. Foods* 38 338–348. 10.1016/j.jff.2017.09.023

[B11] HanT. S.LeanM. E. (2016). A clinical perspective of obesity, metabolic syndrome and cardiovascular disease. *JRSM Cardiovasc. Dis.* 5:2048004016633371. 10.1177/2048004016633371 26998259PMC4780070

[B12] HanT.LvY.WangS.HuT.HongH.FuZ. P. (2019). PPAR γ overexpression regulates cholesterol metabolism in human L02 hepatocytes. *J. Pharmacol. Sci.* 139 1–8. 10.1016/j.jphs.2018.09.013 30554802

[B13] HollowayG. P.BezaireV.HeigenhauserG. J.TandonN. N.GlatzJ. F.LuikenJ. J. (2006). Mitochondrial long chain fatty acid oxidation, fatty acid translocase/CD36 content and carnitine palmitoyltransferase I activity in human skeletal muscle during aerobic exercise. *J. Physiol.* 571 201–210. 10.1113/jphysiol.2005.102178 16357012PMC1805655

[B14] HsuC. C.LaiC. Y.LinC. Y.YehK. Y.HerG. (2018). MicroRNA-27b depletion enhances endotrophic and intravascular lipid accumulation and induces adipocyte hyperplasia in Zebrafish. *Int. J. Mol. Sci.* 19 93–112. 10.3390/ijms19010093 29286302PMC5796043

[B15] HughesT. A. (2006). Regulation of gene expression by alternative untranslated regions. *Trends Genet.* 22 119–122. 10.1016/j.tig.2006.01.001 16430990

[B16] JainS. S.ChabowskiA.SnookL. A.SchwenkR. W.GlatzJ. F.LuikenJ. J. (2009). Additive effects of insulin and muscle contraction on fatty acid transport and fatty acid transporters, FAT/CD36, FABPpm, FATP1, 4 and 6. *FEBS Lett.* 583 2294–2300. 10.1016/j.febslet.2009.06.020 19527715

[B17] JiW.GongL.WangJ.HeH.ZhangY. (2016). hypoxic exercise training promotes apelin/APJ expression in skeletal muscles of high fat diet-induced obese mice. *Protein Pept. Lett.* 24 64–70. 10.2174/0929866524666161111111726 27834140

[B18] JiW.GongL.WangJ.HeH.ZhangY. (2017). Hypoxic exercise promotes apelin/APJ expression in skeletal muscles of high fat diet-induced obese mice. *Protein Pept. Lett.* 24 64–70.2783414010.2174/0929866524666161111111726

[B19] KarbienerM.FischerC.NowitschS.OpriessnigP.PapakC.AilhaudG. (2009). microRNA miR-27b impairs human adipocyte differentiation and targets PPARγ. *Biochem. Biophys. Res. Commun.* 390 247–251. 10.1016/j.bbrc.2009.09.098 19800867

[B20] KayserB.VergesS. (2013). Hypoxia, energy balance and obesity: from pathophysiological mechanisms to new treatment strategies. *Obes. Rev.* 14 579–592. 10.1111/obr.12034 23551535

[B21] KershawE. E.SchuppM.GuanH. P.GardnerN. P.LazarM. A.FlierJ. S. (2007). PPAR γ regulates adipose triglyceride lipase in adipocytes in vitro and in vivo. *Am. J. Physiol. Endocrinol. Metab.* 293 E1736–E1745. 10.1152/ajpendo.00122.2007 17848638PMC2819189

[B22] KongZ.ZangY.HuY. (2014). Normobaric hypoxia training causes more weight loss than normoxia training after a 4-week residential camp for obese young adults. *Sleep Breath* 18 591–597. 10.1007/s11325-013-0922-4 24318688

[B23] KoonenD. P.GlatzJ. F.BonenA.LuikenJ. J. (2005). Long-chain fatty acid uptake and FAT/CD36 translocation in heart and skeletal muscle. *Biochim. Biophys. Acta* 1736 163–180. 10.1016/j.bbalip.2005.08.018 16198626

[B24] LeeM. J.JashS.JonesJ. E.PuriV.FriedS. K. (2019). Rosiglitazone remodels the lipid droplet and britens human visceral and subcutaneous adipocytes ex vivo. *J. Lipid Res.* 60 856–868. 10.1194/jlr.M091173 30782959PMC6446708

[B25] LiY.LiH.HanJ. (2019). Sphingosine-1-phosphate receptor 2 modulates pain sensitivity by suppressing the ROS-RUNX3 pathway in a rat model of neuropathy. *J. Cell Physiol.* 235 3864–3873. 10.1002/jcp.29280 31603252PMC13482701

[B26] LiY.ZhengX.LiuB.YangG. (2010). Regulation of ATGL expression mediated by leptin in vitro in porcine adipocyte lipolysis. *Mol. Cell Biochem.* 333 121–128. 10.1007/s11010-009-0212-4 19626423

[B27] LingQ.SailanW.RanJ.ZhiS.CenL.YangX. (2008). The effect of intermittent hypoxia on bodyweight, serum glucose and cholesterol in obesity mice. *Pak. J. Biol. Sci.* 11 869–875. 10.3923/pjbs.2008.869.875 18814648

[B28] LivakK. J.SchmittgenT. D. (2001). Analysis of relative gene expression data using real-time quantitative PCR and the 2(-Delta C(T)) Method. *Methods* 25 402–408. 10.1006/meth.2001.1262 11846609

[B29] LuoY.WangL.WuX.HouC.LiJ.LvY. (2019). Regulation mechanism of silkworm pupa oil PUFAs on cholesterol metabolism in hepatic cell L-02. *J. Sci. Food Agric.* 100 1418–1425. 10.1002/jsfa.10115 31667852

[B30] MatuJ.O’HaraJ.HillN.ClarkeS.BoosC.NewmanC. (2017). Changes in appetite, energy intake, body composition, and circulating ghrelin constituents during an incremental trekking ascent to high altitude. *Eur. J. Appl. Physiol.* 117 1917–1928. 10.1007/s00421-017-3683-0 28741038PMC5556141

[B31] McGregorR. A.ChoiM. S. (2011). microRNAs in the regulation of adipogenesis and obesity. *Curr. Mol. Med.* 11 304–316. 10.2174/156652411795677990 21506921PMC3267163

[B32] NickersonJ. G.AlkhateebH.BentonC. R.LallyJ.NickersonJ.HanX. X. (2009). Greater transport efficiencies of the membrane fatty acid transporters FAT/CD36 and FATP4 compared with FABPpm and FATP1 and differential effects on fatty acid esterification and oxidation in rat skeletal muscle. *J. Biol. Chem.* 284 16522–16530. 10.1074/jbc.M109.004788 19380575PMC2713524

[B33] NielsenT. S.VendelboM. H.JessenN.PedersenS. B.JørgensenJ. O.LundS. (2011). Fasting, but not exercise, increases adipose triglyceride lipase (atgl) protein and reduces g(0)/g(1) switch gene 2 (g0s2) protein and mrna content in human adipose tissue. *J. Clin. Endocrinol. Metab.* 96 E1293–E1297. 10.1210/jc.2011-0149 21613358

[B34] NielsenT.JessenN.JørgensenJ. O.MøllerN.LundS. (2014). Dissecting adipose tissue lipolysis: molecular regulation and implications for metabolic disease. *J. Mol. Endocrinol.* 52 R199–R122. 10.1530/JME-13-0277 24577718

[B35] OngJ. M.KernP. A. (1989). Effect of feeding and obesity on lipoprotein lipase activity, immunoreactive protein, and messenger RNA levels in human adipose tissue. *J. Clin. Invest.* 84 305–311. 10.1172/JCI114155 2738155PMC303983

[B36] ParkH. Y.JungW. S.KimJ.LimK. (2019). Twelve weeks of exercise modality in hypoxia enhances health−related function in obese older Korean men: a randomized controlled trial. *Geriatr. Gerontol. Int.* 19 311–316. 10.1111/ggi.13625 30788892

[B37] ParkY. K.ParkH. (2012). Differentiated embryo chondrocyte 1 (DEC1) represses PPARγ2 gene through interacting with CCAAT/enhancer binding protein β (C/EBPβ). *Mol. Cells* 33 575–581. 10.1007/s10059-012-0002-9 22610404PMC3887761

[B38] RaynoldsM. V.AwaldP. D.GordonD. F.GutierrezhartmannA.RuleD. C.WoodW. M. (1990). Lipoprotein lipase gene expression in rat adipocytes is regulated by isoproterenol and insulin through different mechanisms. *Mol. Endocrinol.* 4 1416–1422. 10.1210/mend-4-9-1416 2233752

[B39] SchenkS.HorowitzJ. F. (2006). Coimmunoprecipitation of FAT/CD36 and CPT I in skeletal muscle increases proportionally with fat oxidation after endurance exercise training. *Am. J. Physiol. Endocrinol. Metab.* 291 E254–E260. 10.1152/ajpendo.00051.2006 16670153

[B40] SchoonjansK.Peinado−OnsurbeJ.LefebvreA. M.HeymanR. A.BriggsM.DeebS. (1996). PPARalpha and PPARgamma activators direct a distinct tissue−specific transcriptional response via a PPRE in the lipoprotein lipase gene. *EMBO J.* 15 5336–5348.8895578PMC452277

[B41] SelitskyS. R.DinhT. A.TothC. L.KurtzC. L.HondaM.StruckB. R. (2015). Transcriptomic analysis of chronic hepatitis B and C and liver cancer reveals microRNA-mediated control of cholesterol synthesis programs. *mBio* 6 e1500–e1515. 10.1128/mBio.01500-15 26646011PMC4676282

[B42] ShinS. H. (2015). Influences of normobaric hypoxic training on metabolic syndrome and inflammatory risk markers in adult males. *J. Korean Phys. Educ. Assoc. Girls Women* 31 121–134.

[B43] SimsoloR. B.EzzatS.OngJ. M.SaghizadehM.KernP. A. (1995). Effects of acromegaly treatment and growth hormone on adipose tissue lipoprotein lipase. *J. Clin. Endocrinol. Metab.* 80 3323–3328. 10.1210/jcem.80.11.7593431 7593431

[B44] SimsoloR. B.OngJ. M.KernP. A. (1993). The regulation of adipose tissue and muscle lipoprotein lipase in runners by detraining. *J. Clin. Invest.* 92 2124–2130. 10.1172/JCI116813 8227328PMC288390

[B45] SimsoloR. B.OngJ. M.SaffariB.KernP. A. (1992). Effect of improved diabetes control on the expression of lipoprotein lipase in human adipose tissue. *J. Lipid Res.* 33 89–95.1552236

[B46] SinghA. K.AryalB.ZhangX.FanY.PriceN. L.SuárezY. (2018). Posttranscriptional regulation of lipid metabolism by non-coding RNAs and RNA binding proteins. *Semin. Cell Dev. Biol.* 81 129–140. 10.1016/j.semcdb.2017.11.026 29183708PMC5975105

[B47] SteinbergG. R.KempB. E.WattM. J. (2007). Adipocyte triglyceride lipase expression in human obesity. *Am. J. Physiol. Endocrinol. Metab.* 293 E958–E964. 10.1152/ajpendo.00235.2007 17609260

[B48] SutliffR.SearlesC.Jr.HartC.BijliK.GreenD.KangB. Y. (2013). Hypoxia mediates mutual repression between microRNA-27a and PPAR gamma in the Pulmonary Vasculature. *PLoS One* 8:e79503. 10.1371/journal.pone.0079503 24244514PMC3828382

[B49] TomazL. M.BarbosaM. R.FarahnakZ.LagoeiroC. G.MagossoN. S.LavoieJ. M. (2016). GLUT2 proteins and PPARγ transcripts levels are increased in liver of ovariectomized rats: reversal effects of resistance training. *J. Exerc. Nutrition Biochem.* 20 51–55. 10.20463/jenb.2016.06.20.2.7 27508154PMC4977907

[B50] WangR.GuoS.TianH.HuangY.YangQ.ZhaoK. (2019). Hypoxic training in obese mice improves metabolic disorder. *Front. Endocrinol.* 10:527. 10.3389/fendo.2019.00527 31440207PMC6694298

[B51] WesterterpK. R.KayserB. (2006). Body mass regulation at altitude. *Eur. J. Gastroenterol. Hepatol.* 18 1–3. 10.1097/00042737-200601000-00001 16357611

[B52] WorkmanC.BassetF. A. (2012). Post-metabolic response to passive normobaric hypoxic exposure in sedentary overweight males: a pilot study. *Nutr. Metab.* 9 103–111. 10.1186/1743-7075-9-103 23157699PMC3546003

[B53] XinboZ.PriceN. L.Fernández-HernandoC. (2018). Non-coding RNAs in lipid metabolism. *Vascul. Pharmacol.* 114 93–102. 10.1016/j.vph.2018.06.011 29929012PMC6298865

[B54] XuP.GuoH.WangaH.LeeS. C.LiuM.PanY. (2019). Downregulations of placental fatty acid transporters during cadmium-induced fetal growth restriction. *Toxicology* 423 112–122. 10.1016/j.tox.2019.05.013 31152847

[B55] YangL.LuK.WenX.-Y.LiuH.ChenA.-P.XuM.-W. (2012). Jueming Prescription reduces body weight by increasing the mRNA expressions of beta3-adrenergic receptor and uncoupling protein-2 in adipose tissue of diet-induced obese rats. *Chin J. Integr. Med.* 18 775–781. 10.1007/s11655-011-0959-9 22457173

[B56] YangQ.HuangG.TianQ.LiuW.SunX.LiN. (2018). “Living High-training Low” improved weight loss and glucagon-like peptide-1 level in a 4-week weight loss program in adolescents with obesity: a pilot study. *Medicine* 97 e9943–e9952. 10.1097/MD.0000000000009943 29465583PMC5842013

[B57] YingliL.MinhaoX.LianshiF.LiZ.JianfangX.ZihongH. (2014). Promotion of fatty acid oxidation in gastrocnemius of obese rats through 4-week hypoxic living and exercise. *Chinese J. Sports Med.* 33 1060–1068. 10.3969/j.issn.1000-6710.2014.11.005

[B58] YingliL.ZhuL.FengL. (2017). Effects of hypoxic living and exercise training on the miR-27/PPARγ pathway in obese rat liver. *Med. Sci. Sports Exerc.* 49:437 10.1249/01.mss.0000518079.72889.85

[B59] ZhangM.WuJ. F.ChenW. J.TangS. L.MoZ. C.TangY. Y. (2014). MicroRNA-27a/b regulates cellular cholesterol efflux, influx and esterification/hydrolysis in THP-1 macrophages. *Atherosclerosis* 234 54–64. 10.1016/j.atherosclerosis.2014.02.008 24608080

[B60] ZhangY.YangJ.YeJ.GuoQ.WangW.SunY. (2019). Separate and combined associations of physical activity and obesity with lipid-related indices in non-diabetic and diabetic patients. *Lipids Health Dis.* 18:49. 10.1186/s12944-019-0987-6 30755212PMC6371482

[B61] ZhouC.CaoJ.ShangL.TongC.HuH.WangH. (2013). Reduced paraoxonase 1 activity as a marker for severe coronary artery disease. *Dis. Markers* 35 97–103. 10.1155/2013/816189 24167353PMC3774974

[B62] ZhuL.YingliL.FengL. (2018). Study on hypoxia exercise inducing miR-27/PPARγ to regulate fatty acids metabolism in obese rat’s liver. *China Sport Sci. Technol.* 54 115–122. 10.16470/j.csst.201801016

[B63] ZhuL.YingliL.FengL.SuxianZ. (2019). Hypoxia exercise induced miR-27/PPARγ miR-27/PPARγ to regulate fatty acid metabolism in obese rat gastrocnemius. *China Sport Sci.* 39 55–61. 10.16469/j.css.201906007

[B64] ZhuW.ZouB.NieR.ZhangY.LiC. M. (2015). A-type ECG and EGCG dimers disturb the structure of 3T3-L1 cell membrane and strongly inhibit its differentiation by targeting peroxisome proliferator-activated receptor γ with miR-27 involved mechanism. *J. Nutr. Biochem.* 26 1124–1135. 10.1016/j.jnutbio.2015.05.006 26145192

